The article "Investigating Influences of Synthesizing Eco-Friendly Waste-Coir-Fiber Nanofiller-Based Ramie and Abaca Natural Fiber Composite Parameters on Mechanical Properties" was retracted in 2024. Reasons: signs of a paper mill; suspected computer-generated content; unreliable results or conclusions; concerns about the data.

# Investigating Influences of Synthesizing Eco-Friendly Waste-Coir-Fiber Nanofiller-Based Ramie and Abaca Natural Fiber Composite Parameters on Mechanical Properties

**DOI:** 10.1155/2022/6557817

**Published:** 2022-02-04

**Authors:** T. Sathish, Vinayagam Mohanavel, Palanivel Velmurugan, R. Saravanan, T. Raja, M. Ravichandran, Wadi B. Alonazi, Shanmugam Sureshkumar, Atkilt Mulu Gebrekidan

**Affiliations:** ^1^Department of Mechanical Engineering, Saveetha School of Engineering, SIMATS, Chennai 602 105, Tamil Nadu, India; ^2^Centre for Materials Engineering and Regenerative Medicine, Bharath Institute of Higher Education and Research, Selaiyur, Chennai 600073, Tamil Nadu, India; ^3^Department of Mechanical Engineering, Vel Tech Rangarajan Dr. Sakunthala R&D Institute of Science and Technology, Chennai 600062, India; ^4^Department of Mechanical Engineering, K. Ramakrishnan College of Engineering, Trichy 621112, Tamil Nadu, India; ^5^Health Administration Department, College of Business Administration, King Saud University, PO Box 71115, Riyadh 11587, Saudi Arabia; ^6^Department of Animal Resources Science, Dankook University, 119,Dandae-ro, Cheonan,31116, Republic of Korea; ^7^Department of Mechanical Engineering, Faculty of Mechanical Engineering, Arba Minch Institute of Technology (AMIT), Arba Minch University, Addis Ababa, Ethiopia

## Abstract

Clean technology-based natural fiber composite fabrication is the prime aim of this piece of research. Natural fibers highly replace metal usage in industries and automobile, marine, medical applications, and so on. Vast amounts of natural fibers are freely available in all areas. In this research, work nanofiller material such as nano form waste coir fiber is collected from used car seat. The 10 wt.% of nanofiller material is added to the preparation of natural nanocomposites (ramie and abaca fiber). Hybrid composites are fabricated with the influence of different process parameters, namely, fiber weight percentage (20 wt.%, 30 wt.%, 40 wt.%, and 50 wt.%), NaOH action % (4%, 6%, 8%, and 10%), compression pressure (9 MPa, 12 MPa, 15 MPa, and 18 MPa), and temperature (100°C, 120°C, 140°C, and 160°C). Furthermore, the strength of this hybrid composite has analyzed by conducting flexural, impact, and shore hardness tests. These tests have provided the influence of selected parameters and their effects on the results of experimental work. In the flexural analysis, 6% of NaOH action has offered maximum flexural strength of the specimens. Correspondingly in the impact test, 30 wt.% of fiber is produced higher impact strength. Finally, applying 15 Mpa of compression pressure records the maximum shore hardness.

## 1. Introduction

Nowadays, the environment-friendly composite invention is most indispensable. The utilization of waste is encouraged by clean technology. This research focuses on the used (waste) coir fibers in nano form as filler for fabricating the natural fiber composites. Many industries like to use natural fibers for their production parts and encourage research-oriented analysis in utilizing natural fiber. Composite fabrication is one of the novelty work in engineering fields and also in science-applied projects. Compared to metal matrix composites, polymer matrix composites are light in weight and used in different automobile, aircraft, and marine applications. Recently, the marine boats had produced by fiber amalgamation to ensure the lightweight of the boat structure [1]. In contrast to synthetic fiber, the guaruman fiber is one of the cheapest fibers and is extremely used in all applications. This fiber is highly applicable in biomedical applications; it possesses high strength and biodegradability and is easy to renewable [2]. The flax fiber quality and its strength have been analyzed through the tensile test. The tensile strength is highly improved, as the maximum tensile strength has been found (865 MPa) by using flax fiber with epoxy resin [3]. Natural fibers are replaced glass fiber in several applications based on the properties such as physical and mechanical. This natural fiber is eco-friendly, low cost, and biodegradable. Fly ash is the best filler material in all-natural fibers, especially in banana fiber with reinforced polyester. Various percentage of fly ash has influenced to improve the mechanical strength, namely tensile, flexural, and affect. Adding fly ash filler material is to reduce the moisture absorption resistance of the natural fiber composites. This result has been found by using a scanning electron microscope [4]. Different natural fibers, namely, birch, palm, and eucalyptus fibers, produce the hybrid composites with the help of epoxy resin. Composites are prepared by using resin transfer moulding and moulded fiber making practice amalgamation. Higher tensile stress has been registered (45.28 MPa) by using eucalyptus reinforced epoxy composites. Similarly, in bending stress, the maximum bending stress of 79.92 MPa has been observed [5]. Based on the industrial applications and high demand, industrialists have turned towards consuming natural fibers instead of synthetic polymers. Most of the automotive and wood industries focus on natural fibers, namely, jute, hemp, sisal, kenaf, bamboo, cotton, flax, abaca, coir, and so on. Now, research has moved to analyze the strength of the natural fibers in contrast to synthetic fibers [6]. Chemical treatment of the fibers is enhanced the mechanical properties; few investigations are concentrated on the chemical treatment of the fibers. Natural fibers of jute, sisal, and kenaf have been considered for preparing hybrid composites using epoxy resin. The composites are prepared by implementing of hand lay-up method. In hybrid composites preparation, the mixing range of resigning and fibers are 30% and 70%, respectively. Always the mechanical tests have been conducted with consideration of ASTM standards. In each mechanical test, the fracture analysis has conducted through scanning electron microscopy (SEM) [7]. Sodium hydroxide (NaOH) treatment is excellent for improving the mechanical properties of banana fibers. The different percentages have been considered such as 1%, 3%, 5%, 7%, and 9% of NaOH. Chemically treated and untreated banana fibers have been tested by applying Fourier-transform infrared spectrometry (FTIR) to categorize the chemical compounds present in the fibers. The morphological investigation has been carried out by using of scanning electron microscope [8]. Biocomposites of the banana-pineapple leaf are fabricated using epoxy resin. The banana-pineapple fibers have been used in different weight percentages such as 30 wt.%, 40 wt.%, and 50 wt.%. They analyzed the strength of the composites through the three-point flexural test. From this test, the results have concluded the 40 wt.% of fibers offered the maximum flexural strength of the composites. Increasing both compaction pressure and packing of fibers are introduced to the failure of the composites. The thermal steadiness of the composites has been analyzed by applying thermal gravimetric analysis (TGA) and dynamic mechanical analysis (DMA) tests [9]. This research work is planned and executed to analyze the mechanical strength of the nano-sized waste-coir-fiber-filled natural-fiber polymer-matrix composites. Two natural fibers, namely, ramie and abaca, have been used for the preparation of the composites. Epoxy resin is taken to prepare the composites with different parameters that are accounted. The outcome of this research work has focused on flexural strength, impact strength, and shore hardness.

## 2. Materials and Methods

The two natural fibers were procured for this investigation, namely, ramie and abaca; both are high strength and high stiffness fibers [10–12]. The ramie fiber was purchased from the Fiber Region, Chennai, and the abaca fiber is purchased from Vruksha Composites, Chennai. Both the fibers were procured in kilogram; Figure 1 illustrates the natural fibers of ramie and abaca. Waste coir fibers have collected from the used sofa, bed, and car seat as a sample, and they were brominated in a bath of saturated bromine water. Then they were treated with the use of stannous chloride solution as suggested by [13]. The treated waste coir fibers were dried well. The processed waste coir fibers grounded well to less than 30 nm size. The ball mill has been used to mix the waste coir nanofibers with the resin to obtain uniform distribution of nanofillers.

Natural fibers are cleaned well, and using compression molding, the hybrid composites are produced with the influence of different process parameters [14–16]. The Taguchi route was implemented to find the superior mechanical properties, namely, flexural strength, impact strength, and shore hardness of the composites. Mostly, the composites are produced by using a polymer matrix. This matrix is commonly used for producing composites with the assistance of resin solution. Using resin matrix, the listed properties of the composites are identified such as high strength, little amount of shrinkage, improved adhesion properties, good electrical property, chemical resistance, and low toxicity.

### 2.1. Experimental Procedure

In the initial stage, the fibers are cleaned thoroughly with the help of running water; furthermore, the fibers are processed by chemical treatment. This work considered the chemical treatment with the influence of sodium hydroxide solution. Chemical action was carried out with a different percentage of using NaOH solution such as 4%, 6%, 8%, and 10%. Using distilled water in a beaker, mix different weight percentages of NaOH solution, such as 4 wt. percent, 6 wt. percent, 8 wt. percent, and 10 wt. percent. This process was used to remove the waste substance; wax segment and a few of the hemicelluloses were present in the fibers for improving the crystalline property of the matrix composites [17–19]. The chemical processing is maintained at room temperature with 2 hrs of soaking time for complete cleaning of the fibers. After chemical treatment, the fibers were again washed and permitted to dry condition; furthermore, the fibers are heated well in the oven. The heating process was carried out with a temperature of 80°C and for a period of 4 h [20]. The chemical treatment increased the chemical composition of the fibres, which had 40.3 percent cellulose, 32.5 percent hemicelluloses, and 20.0 percent total lignin before chemical treatment. After chemical treatment, the chemical composition of the fibers is altered such as 82.4% of cellulose, 5.2% of hemicelluloses, and 8.4% of total lignin. Before conducting chemical treatment, the density of the fiber is 1.17 g/cm^3^; after chemical treatment, the density of the fiber is 1.29 g/cm^3^. All the fibers were hacked for the length of 10 mm uniformly; blended ramie and abaca with different weight percentages (20 wt.%, 30 wt.%, 40 wt.%, and 50 wt.%) were placed in the mould. The mould was made of steel material; the raw mould specimen was prepared under the dimension of 250 mm × 250 mm × 5 mm [21–24]. Epoxy resin was poured as the matrix material into the blended fiber in the steel mould at the required weight percentage. The compression process has been carried out with different pressure ranges such as 9 MPa, 12 MPa, 15 MPa, and 18 MPa. The temperature was maintained during the compression process such as 100°C, 120°C, 140°C, and 160°C. Fabrication of fibers was concentrated to the different parameters with the concern of Taguchi analysis; Table 1 presented the process parameters for fabrication of hybrid composites. The density of the prepared composite is 1.218 g/cm^3^; similarly, the void fraction is observed (0.612%).

The flexural test was conducted through a three-point loader arrangement in the universal testing machine (UTM) with ASTM standard (ASTM D790) as shown in Figure 2. The UTM (Universal Grip Company, Salem) has 5 KN capacity and load cell arrangements [25]. The operating speed for the flexural test was 2 mm/min for the polymer composite material. A flexural test specimen was prepared under the dimensions of 150 mm × 15 mm × 5 mm [26–28].

Impact test was conducted by using of impact tester with Charpy mode; the ASTM D 256 standard procedure was applied for the impact test [29]. The dimensions of the impact test were prepared such as 50 mm × 10 mm × 5 mm; model of the impact test machine was ASR-XJJ-11. The pendulum energy range was 2.75 J, 5.5 J, and 11 J, and the test angle was 150°.  Figure 3 illustrates the image of impact test specimens [30].

Hardness is one of the mechanical properties that has to ensure the resistance to indentation; normally, the hardness of the MMCs was measured by Rockwell or Brinell hardness tester [31]. This investigation considers the shore D hardness tester for measuring the hybrid composites (Linear Instruments, Chennai). Shore D hardness was applied to take hardness reading from the composites in multiple numbers and finally average it (see Figure 4).

## 3. Results and Discussion

### 3.1. Flexural Test

Table 2 presented the outline of flexural strength with the influence of parameters; the highest flexural strength was found (78.29 MPa). Maximum flexural strength was reached by involving a different set of parameters such as 50 wt.% of fiber, 6% of the chemical action of NaOH solution, 15 MPa of compression pressure, and 100°C temperature.

Tables 3 and 4 represented the response tables for means and S/N ratio of the flexural strength analysis. Rank order was concluded as the highest influence factor in the flexural strength test. Chemical treatment such as the NaOH action parameter was extremely influenced and continued by compression temperature, fiber weight percentage, and compression pressure. From the flexural test, the optimal parameters were attained such as 50 wt.% of fiber, 6% of NaOH action, 9 MPa of compression pressure, and 130°C of compression temperature.

Figures 5 and 6 illustrate both main effect plots for means and S/N ratio of flexural strength, respectively. In fiber weight percentage, the increasing trends of weight percentage increase the flexural strength; initially, the 20 wt.% of fiber offered low flexural strength. The maximum flexural strength was obtained by influencing 50 wt.% of fiber. From the chemical treatment, the 6% of NaOH action has to be produced the maximum flexural strength; continually increasing the NaOH percentage can reduce the flexural strength.

Low compression pressure (9 MPa) offered excellent flexural strength; growing the compression pressure can decrease the flexural strength. The low temperature of the process provided low flexural strength; maximum temperature levels such as 130°C recorded extreme flexural strength.

Figure 7 shows the interval plot of flexural strength analysis; this plot highly enlightens all parameters influences in a single hand. From this plot, the maximum flexural strength was obtained (78.29 MPa) with an influence of 50 wt.% of fiber, 6% of NaOH action, 15 MPa of compression pressure, and 100°C of temperature.

Figures 8–11 demonstrate the surface plot for flexural strength analysis.  Figure 8 presented the correlation between fiber weight percentage and NaOH action; in this relation, the 50 wt.% of fiber and 6% of NaOH action were registered as the highest flexural strength.  Figure 9 exemplified the relationship between compression pressure and NaOH action; it was concluded that the maximum flexural strength was attained by the way of 9 MPa of compression pressure and 6% of NaOH action.  Figure 10 illustrates the connection between temperature and compression pressure; this informs that higher flexural strength was recorded by100°C of temperature and 15 MPa of compression pressure.  Figure 11 shows the association between fiber weight percentage and temperature; this correlation proved that 30 wt.% of fiber and 130°C of temperature offered excellent flexural strength.

### 3.2. Impact Strength

Table 5 illustrates the summarization of impact strength with the influence of parameters; the maximum impact strength was recorded (26.58 kJ/m^2^). The higher impact strength was achieved by the way of concerning of parameters, namely, 50 wt.% of fiber, 4% of the chemical action of NaOH solution, 18 MPa of compression pressure, and 110°C of temperature.

Tables 6 and 7 present the response tables for means and S/N ratio of the impact strength investigation. In all these analyses, the rank order was notified of the most manipulated factors in the impact strength test. Among all four parameters, the fiber weight percentage was highly influenced, followed by compression pressure, NaOH action, and compression temperature. In the impact test, optimal parameters were accomplished such as 30 wt.% of fiber, 6% of NaOH action, 15 MPa of compression pressure, and 130°C of compression temperature.

Figure 12 illustrates the main effect plot for means, and Figure 13 shows the main effect plot for the S/N ratio of impact strength. Relating to fiber weight percentage, the maximum impact strength was recorded by the influence of 30 wt.% of fiber; by further increasing the fiber weight percentage, the impact strength was reduced. Considering the NaOH action parameter, the 6% of NaOH offered maximum impact strength that continually increases the NaOH action; the strength has to be reduced. Compression pressure of 15 MPa offered maximum impact strength; low compression pressure produced the minimum strength. During compression, the 130°C of temperature offered the maximum impact strength.

Figure 14 illustrates the interval plot of impact strength examination; this plot extremely informed every parameter's influences in the same plot for easy to understand. From this plot, it is clear that the highest impact strength was registered as 26.58 kJ/m^2^. The maximum impact strength was attained with the influence of 50 wt.% of fiber, 4% of NaOH action, 18 MPa of compression pressure, and 110°C of temperature.

Figures 15–18 reveal the 3D Trajectory plot for impact strength investigation.  Figure 15 illustrates the connection between fiber weight percentage and NaOH action; for this relation, the 50 wt.% of fiber and 4% of NaOH action were recorded as the maximum impact strength.  Figure 16 illustrates the correlation between compression pressure and NaOH action; it is resulted from the greatest impact strength that was obtained by the way of 15 MPa of compression pressure and 6% of NaOH action.  Figure 17 shows the link between temperature and compression pressure; this report to superior impact strength was registered by 110°C of temperature and 18 MPa of compression pressure.  Figure 18 shows the relationship between fiber weight percentage and temperature; this connection confirmed the 50 wt.% of fiber and 110°C of temperature that offered exceptional impact strength.

### 3.3. Shore D Hardness

Table 8 presents the shore D hardness with the influence of parameters; in this investigation, the highest shore D hardness was 72 HD. It was achieved in the twelfth experimental run from L16 OA. The greater shore D hardness was accomplished parenthetically by relating to parameters specifically 40 wt.% of fiber, 10% of the chemical action of NaOH solution, 12 MPa of compression pressure, and 100°C of temperature.

Tables 9 and 10 illustrate the response tables for means and S/N ratio of the shore D hardness test examination. From all these studies, the rank order was informed the majority influence factor in the shore D hardness test. Among all four parameters, the compression pressure was extremely influenced in contrast to the remaining factors, followed by fiber weight percentage, compression pressure, compression temperature, and NaOH action. From the shore D hardness test, the optimal parameters were obtained such as 40 wt.% of fiber, 10% of NaOH action, 15 MPa of compression pressure, and 100°C of compression temperature.

Figure 19 presents the main effect plot for means, and Figure 20 demonstrates the main effect plot for the S/N ratio of shore D hardness. Connecting to fiber weight percentage, the highest shore D hardness was registered by the influence of 40 wt.% of fiber; by further increasing the fiber weight percentage, the shore D hardness was reduced. Regarding the NaOH action parameter, 10% NaOH generated outstanding hardness values. Increasing compression pressure such as 9 MPa to15 MPa offered maximum hardness values; 9 MPa of low compression pressure reduces the hardness values. At the time of compression, the minimum level of 100°C of temperature provided the hardness of the composites [32–39].

Figure 21 represents the interval plot of shore D hardness inspection; this plot exceptionally informed the influence of each parameter in the same plot for simple to understand. From this plot, it is clear that the maximum shore D hardness was found (72 HD). This maximum shore D hardness was obtained with the influence of 40 wt.% of fiber, 10% of NaOH action, 12 MPa of compression pressure, and 100°C of temperature.

Figures 22–25 show the contour plot for shore D hardness analysis.  Figure 22 shows the correlation between fiber weight percentage and NaOH action; for this interaction, the 30 wt.% of fiber and 10% of NaOH action produced the maximum hardness values.  Figure 23 illustrates the relationship between compression pressure and NaOH action; it was notified that the maximum shore D hardness was obtained incidentally of 12 MPa of compression pressure and 10% of NaOH action.  Figure 24 represents the connection between temperature and compression pressurea temperature of 100°C and a compression pressure of 12 MPa resulted in higher hardness.  Figure 25 demonstrates the correlation of fiber weight percentage and temperature; this correlation confirmed that the 40 weight percentage of fiber and 100°C of temperature presented excellent hardness values.

Figure 26 illustrates the 2D and 3D profilometric images of the flexural test specimen. The SEM image was converted into a profilometric image; the uneven blending of epoxy resin with fiber was represented in pink color. In Figure 27, the epoxy resin was homogeneously mixed into the fibers; it can be reflected in greenish yellow color in the impact test samples. Both the images were concluded the blending of fiber and epoxy resin in a uniform manner.

## 4. Conclusion

The environment-friendly clean technology-based natural fiber composite fabrication was focused on in this piece of research. The cheap and best natural fibers and nanofillers from waste coir are utilized to fabricate compression moulding. The compression moulding parameters such as temperature and compression pressures were varied at four levels. The fiber quality by NaOH treatment as well as quantity of fiber content also varied at four levels. The nano-sized treated waste coir filler was utilized at a fixed weight percentage. The widely and cheaply available natural fibers such as ramie and abaca were used to prepare the natural fiber composites effectively in the matrix of epoxy resin. The composite samples were fabricated as per Taguchi design of experiment L16. The samples were tested for mechanical characteristics such as flexural strength, impact strength, and shore hardness; the findings of this investigation were summarized below:

- From the flexural analysis, the highest flexural strength was found (78.29 MPa). Maximum flexural strength was attained by concerning different sets of parameters such as 50 wt.% of fiber, 6% of the chemical action of NaOH solution, 15 MPa of compression pressure, and 100°C of temperature. In the flexural test, the optimal parameters were found such as 50 wt.% of fiber, 6% of NaOH action, 9 MPa of compression pressure, and 130°C of compression temperature.
- In the impact strength analysis, the maximum impact strength was registered (26.58 kJ/m^2^). The superior impact strength was accomplished by relating to different parameters, namely, 50 wt.% of fiber, 4% of the chemical action of NaOH solution, 18 MPa of compression pressure, and 110°C of temperature. The impact test concluded that the optimal parameters were obtained such as 30 wt.% of fiber, 6% of NaOH action, 15 MPa of compression pressure, and 130°C of compression temperature.
- From the shore hardness analysis, the maximum shore D hardness was found (72 HD). The enhanced shore D hardness was obtained parenthetically of involving the parameters, specifically 40 wt.% of fiber, 10% of the chemical action of NaOH solution, 12 MPa of compression pressure, and 100°C of temperature. In shore D hardness test, the optimal parameters were found such as 40 wt.% of fiber, 10% of NaOH action, 15 MPa of compression pressure, and 100°C of compression temperature.

## Figures and Tables

**Figure 1:** Natural fibers: (a) ramie fiber and (b) abaca fiber.

**Figure 2:** Three-point bending test arrangement with specimens.

**Figure 3:** Impact test specimens.

**Figure 4:** Shore D hardness specimen.

**Figure 5:** Main effect plot for means to flexural strength.

**Figure 6:** Main effect plot for S/N ratio to flexural strength.

**Figure 7:** Interval plot used in flexural strength analysis.

**Figure 8:** Flexural strength: surface plot of fiber weight percentage and NaOH action.

**Figure 9:** Flexural strength: surface plot of compression pressure and NaOH action.

**Figure 10:** Flexural strength: surface plot of temperature and compression pressure.

**Figure 11:** Flexural strength: surface plot of fiber weight percentage and temperature.

**Figure 12:** Main effect plot for means to impact strength.

**Figure 13:** Main effect plot for means to impact strength.

**Figure 14:** Interval plot used in impact strength analysis.

**Figure 15:** Impact strength: 3D trajectory plot of fiber weight percentage and NaOH action.

**Figure 16:** Impact strength: 3D trajectory plot of compression pressure and NaOH action.

**Figure 17:** Impact strength: 3D trajectory plot compression pressure.

**Figure 18:** Impact strength: 3D trajectory plot of temperature and fiber weight percentage and temperature.

**Figure 19:** Main effect plot for means to shore D hardness.

**Figure 20:** Main effect plot for S/N ratio to shore D hardness.

**Figure 21:** Interval plot of shore D hardness inspection.

**Figure 22:** Shore D hardness: contour plot of fiber weight percentage and NaOH action.

**Figure 23:** Shore D hardness: contour plot of compression pressure and NaOH action.

**Figure 24:** Shore D hardness: contour plot of temperature and compression pressure.

**Figure 25:** Shore D hardness: contour plot of fiber weight percentage and temperature.

**Figure 26:** 2D and 3D profilometric image of the flexural test specimen.

**Figure 27:** 2D and 3D profilometric image of the impact test specimen.

**Table 1:** Process parameters for fabrication of hybrid composites.

Factors	Level 1	Level 2	Level 3	Level 4
Fiber (wt.%)	20	30	40	50
NaOH action (%)	4	6	8	10
Compression pressure (MPa)	9	12	15	18
Temperature (°C)	100	120	140	160

**Table 2:** Outline of Flexural strength with the influence of parameters.

Exp. runs	Fiber (wt.%)	NaOH action (%)	Compression pressure (MPa)	Temperature (°C)	Flexural strength (MPa)	S/N ratio
1	20	4	9	100	68.96	36.7719
2	20	6	12	110	70.25	36.9329
3	20	8	15	120	58.36	35.3223
4	20	10	18	130	72.45	37.2008
5	30	4	12	120	68.36	36.6960
6	30	6	9	130	77.24	37.7568
7	30	8	18	100	65.75	36.3579
8	30	10	15	110	72.89	37.2534
9	40	4	15	130	70.59	36.9749
10	40	6	18	120	65.87	36.3738
11	40	8	9	110	62.49	35.9162
12	40	10	12	100	69.34	36.8197
13	50	4	18	110	70.83	37.0043
14	50	6	15	100	78.29	37.8741
15	50	8	12	130	64.28	36.1615
16	50	10	9	120	73.21	37.2914

**Table 3:** Response table for means (flexural strength).

Level	Fiber (wt.%)	NaOH action (%)	Compression pressure (MPa)	Temperature (°C)
1	67.50	69.69	70.47	70.58
2	71.06	72.91	68.06	69.11
3	67.07	62.72	70.03	66.45
4	71.65	71.97	68.72	71.14
Delta	4.58	10.19	2.42	4.69
Rank	3	1	4	2

**Table 4:** Response table for signal-to-noise ratios (flexural strength); larger is better.

Level	Fiber (wt.%)	NaOH action (%)	Compression pressure (MPa)	Temperature (°C)
1	36.56	36.86	36.93	36.96
2	37.02	37.23	36.65	36.78
3	36.52	35.94	36.86	36.42
4	37.08	37.14	36.73	37.02
Delta	0.56	1.29	0.28	0.60
Rank	3	1	4	2

**Table 5:** Summarization of impact strength with the influence of parameters.

Exp. runs	Fiber (wt.%)	NaOH action (%)	Compression pressure (MPa)	Temperature (°C)	Impact strength (kJ/m^2^)	S/N ratio
1	20	4	9	100	8.96	19.0462
2	20	6	12	110	14.38	23.1552
3	20	8	15	120	18.34	25.2680
4	20	10	18	130	12.75	22.1102
5	30	4	12	120	19.62	25.8540
6	30	6	9	130	22.45	27.0243
7	30	8	18	100	24.21	27.6799
8	30	10	15	110	19.87	25.9640
9	40	4	15	130	16.37	24.2810
10	40	6	18	120	13.08	22.3322
11	40	8	9	110	9.47	19.5270
12	40	10	12	100	11.47	21.1913
13	50	4	18	110	26.58	28.4911
14	50	6	15	100	22.39	27.0011
15	50	8	12	130	17.67	24.9447
16	50	10	9	120	14.73	23.3641

**Table 6:** Response table for means (impact strength).

Level	Fiber (wt.%)	NaOH action (%)	Compression pressure (MPa)	Temperature (°C)
1	13.61	17.88	13.90	16.76
2	21.54	18.07	15.79	17.31
3	12.60	17.42	19.24	16.44
4	20.34	14.71	19.16	17.57
Delta	8.94	3.37	5.34	1.13
Rank	1	3	2	4

**Table 7:** Response table for signal-to-noise ratios (impact strength); larger is better.

Level	Fiber (wt.%)	NaOH action (%)	Compression pressure (MPa)	Temperature (°C)
1	22.39	24.42	22.24	23.73
2	26.63	24.88	23.79	24.28
3	21.83	24.35	26.63	24.20
4	25.95	23.16	25.13	24.59
Delta	4.80	1.72	3.39	0.86
Rank	1	3	2	4

**Table 8:** The shore D hardness with the influence of parameters.

Exp. runs	Fiber (wt.%)	NaOH action (%)	Compression pressure (MPa)	Temperature (°C)	Shore D hardness (HD)	S/N ratio
1	20	4	9	100	58	35.2686
2	20	6	12	110	62	35.8478
3	20	8	15	120	64	36.1236
4	20	10	18	130	60	35.5630
5	30	4	12	120	63	35.9868
6	30	6	9	130	59	35.4170
7	30	8	18	100	70	36.9020
8	30	10	15	110	71	37.0252
9	40	4	15	130	68	36.6502
10	40	6	18	120	65	36.2583
11	40	8	9	110	61	35.7066
12	40	10	12	100	72	37.1466
13	50	4	18	110	70	36.9020
14	50	6	15	100	67	36.5215
15	50	8	12	130	62	35.8478
16	50	10	9	120	59	35.4170

**Table 9:** Response table for means (shore D hardness).

Level	Fiber (wt.%)	NaOH action (%)	Compression pressure (MPa)	Temperature (°C)
1	61.00	64.75	59.25	66.75
2	65.75	63.25	64.75	66.00
3	66.50	64.25	67.50	62.75
4	64.50	65.50	66.25	62.25
Delta	5.50	2.25	8.25	4.50
Rank	2	4	1	3

**Table 10:** Response table for signal-to-noise ratios (shore D hardness); larger is better.

Level	Fiber (wt.%)	NaOH action (%)	Compression pressure (MPa)	Temperature (°C)
1	35.70	36.20	35.45	36.46
2	36.33	36.01	36.21	36.37
3	36.44	36.14	36.58	35.95
4	36.17	36.29	36.41	35.87
Delta	0.74	0.28	1.13	0.59
Rank	2	4	1	3

## Data Availability

The data used to support the findings of this study are included in the article. Should further data or information be required, they can be obtained from the corresponding author upon request.
